The article "Tandem Mass Tag Analysis of the Effect of the Anterior Cingulate Cortex in Nonerosive Reflux Disease Rats with Shugan Jiangni Hewei Granules Treatment" was published in 2022. Journal: Comput Math Methods Med.

# Tandem Mass Tag Analysis of the Effect of the Anterior Cingulate Cortex in Nonerosive Reflux Disease Rats with Shugan Jiangni Hewei Granules Treatment

**DOI:** 10.1155/2022/8104337

**Published:** 2022-07-30

**Authors:** Tianzuo Wang, Jing Li, Yuebo Jia, Jiaqi Zhao, Meijun He, Guang Bai

**Affiliations:** ^1^Liaoning University of Traditional Chinese Medicine, Shenyang, Liaoning 110847, China; ^2^Department of Gastroenterology, Affiliated Hospital of Liaoning University of Traditional Chinese Medicine, Shenyang, Liaoning 110033, China

## Abstract

**Objective:**

The current study aims to analyze the improvement mechanism of visceral hypersensitivity (VH) and targets of Shugan Jiangni Hewei granules (SJHG) for nonerosive reflux disease (NERD) treatment as well as to offer an experimental foundation for its clinical use.

**Methods:**

Healthy male Sprague–Dawley rats (*n* = 36) were acquired in the current study that was further split into three groups: blank, model, and drug (SJHG). Subsequently, differentially expressed proteins and bioinformatics analysis were performed on the collected tissue samples acquired from the anterior cingulate cortex of the model and SJHG rat groups using a tandem mass tag- (TMT-) based proteomics. Eventually, the obtained data from the bioinformatic analysis was further verified through western blotting.

**Results:**

From the bioinformatics analysis, only 64 proteins were differentially expressed between the NC and SJHG groups. These molecules were found to be highly expressed in immunological response and neural signal transmission. Finally, we confirmed three therapeutic targets of SJHG, namely, kininogen 1 (Kng1), junctional adhesion molecule A (JAM-A), and the PI3K/Akt signaling pathway.

**Conclusions:**

SJHG is effective in treating VH, Kng1 and JAM-A may be therapeutic targets of SJHG, and the therapeutic mechanism of SJHG may be realized by influencing immune response or transmission of neural signals.

## 1. Introduction

Gastroesophageal reflux disease (GERD) is described as a chronic condition via the Montreal Consensus report in which the reflux of stomach contents into the oesophagus causes a variety of linked symptoms, the most prominent of which are acid reflux and heartburn [1]. GERD is very common in the community, and the incidence of GERD in China is 8.2%–17.3% [2, 3]. Current information on the phenotypic manifestations of GERD indicates that there are two main phenotypic manifestations—namely, erosive and nonerosive reflux disease (NERD) [4]. NERD also has symptoms such as acid reflux and heartburn; however, no erosion or damage to the esophageal mucosa was observed with traditional endoscopy [5]. It is worth noting that recent studies found that esophageal-dilated intercellular spaces (DIS) could be found in NERD patients under electron microscopy [6]. Clinically, the incidence of NERD is significantly higher than that of the other subtype of GERD, accounting for about 70% of GERD cases [7, 8]. Visceral hypersensitivity (VH) is a phenomenon in which the threshold of uncomfortable visceral stimulation or abnormal pain decreases, or the viscera reacts strongly to traumatic stimulation or demonstrates discomfort with physiological stimulation, which is considered to be an important pathological mechanism of NERD [9]. NERD is often accompanied by psychological symptoms such as anxiety, depression, and panic, which are thought to be related to the sensory enhancement triggered by the central mechanism of VH [10, 11]. Interestingly, the effect is mutual; several studies have found that irritability, anxiety, and other psychological effects of long-term stimulation can make the central nervous system (CNS)—including the anterior cingulate gyrus, amygdala, insula, hypothalamus, prefrontal cortex, and other brain areas—show abnormal activation, thereby aggravating the degree of VH [12, 13]. Mechanical stimulation of the colon results in persistent hyperactivation of the middle cingulate cortex; in acute colitis, downregulation of anterior cingulate cortex excitability successfully attenuates visceral hypersensitivity, anxiety-like behaviors, and visceral motor response [14]. CNS neurons in a VH state demonstrated increased release of a variety of neurotransmitters, which are mostly encapsulated in vesicles for transport [15]. In addition, c-fos is a nucleophosmin whose positive expression is highly correlated with visceral sensitivity and is considered a biomarker of VH [16].

NERD is classified under the umbrella of “swallowing acid” conditions by traditional Chinese medicine (TCM) theory, and its pathogenesis has been defined by liver qi stagnation, stomach discomfort, and adverse stomach qi rising [17]. Clinical manifestations of NERD include belching, throat discomfort, liver depression, and qi stagnation as the primary symptoms. Therefore, Shugan Jiangni Hewei granules (SJHG) were produced as a possible therapeutic agent according to the principle of “disperse and rectify the depressed liver-energy, harmonize the stomach, and regulate vital energy.” Its ingredients include 9 g of Radix Bupleuri (Chaihu), 12 g of Arum Ternatum Thunb (BanXia), 9 g of Chuanxiong Rhizoma (ChuanXiong), 12 g of Aurantii Fructus (ZhiQiao), 12 g of Citrus Reticulata (ChenPi), 9 g of licorice (GanCao), 9 g of Cyperi Rhizoma (XiangFu), 9 g of Inulae Flos (XuanFuHua), 30 g of Reddle (DaiZheShi), and 10 g of Scutellariae Radix (HuangQin) [18]. In our previous study, compared to standard drug therapy, we found that SJHG not only more effectively improved the symptoms of acid reflux and heartburn in NERD patients but also significantly reduced the scores of anxiety and depression in patients [19]. As a result, it was hypothesized that SJHG may cause a decrease in neurosensitivity in NERD patients' brains. Differentially expressed molecules in the anterior cingulate gyrus were screened via tandem mass tag- (TMT-) labeled proteomics and the activities of these proteins were examined using bioinformatics tools to investigate the possible mechanism of SJHG in enhancing VH in NERD. Eventually, a western blot experiment was performed to confirm essential molecules. The objective of this research was to discover how VH causes NERD in the brain, as well as its possible treatment targets.

## 2. Materials and Methods

### 2.1. SJHG Preparation

SJHG is composed of 11 herbal medicines (see Table 1). Tian Jiang Pharmaceutical Co. Ltd. (Jiangsu, China) supplied all of the herbs used in this composition study. The firm produced inspection report certifications for all herbs, and all fulfilled the *Chinese Pharmacopoeia's* criteria (2020).

### 2.2. Animals

The experimental animal center of Liaoning University of Traditional Chinese Medicine (no. 210726211100566367), China, provided 40 male Sprague–Dawley rats (of particular pathogen–free grade, weighing 250 ± 20 g) for this study. The dietary intake of these rats was set as 25 g/day, with unrestricted drinking water access at the experimental animal facility, which had a temperature range of 22°C–25°C, a relative humidity range of 45–60%, and a light cycle of 12/12 hours. All of the methods for the experiments were carried out in accordance with a plan authorized by the Experimental Animal Ethics Committee of Liaoning University of Traditional Chinese Medicine (animal ethics no. 21000042021049). Eventually, the rats were divided into three research groups randomly after the adaptive feeding for one week. The normal control (NC) group rats were fed generally for four weeks and then received intraperitoneal injections of normal saline on the 14^th^ day of the experiment and a gavage of 1.5 mL normal saline in the last two weeks of the experiment. There was no additional intervention in this group. Separately, rats in a NERD group were treated to chronic random stress for 21 days and were then exposed to 1–2 forms of stress stimulation each day following adaptive feeding for 1 week, as described below: (1) Fasting for <20 h, (2) 17 h of water cutoff, (3) swimming for 5 min at 4°C, (4) 17 h 45° cage tilt, (5) shaking stress (high-speed shaking) for 10 min, (6) binding stress for 2 h, (7) wet cushion material exposure (200 mL of water and 100 g of sawdust) for 5 h, or (8) tail-clamping for 2 min. It was opted to inject ovalbumin (#A8040; Solarbio, Beijing, China) and aluminum hydroxide adjuvant (#77161; Thermo Fisher Scientific, Waltham, MA, USA) mixture with a 1 : 2 ratio intraperitoneally on day 14 of the experiment. In the NERD group, from week 3, normal saline was administered intragastrically for 14 days. On day 29, esophageal acid perfusion was performed. The methods of esophageal acid infusion were as follows: the rats were fasted for 24 h before acid infusion, and each rat's head was raised 20°–30° in the supine position after anesthesia with urethane (IE0570; solarbio, Beijing, China). The abdominal wall was cut open to expose the stomach wall, and a small round hole was cut near the cardia, through which the drainage tube was placed to collect fluid from the perfusion. During the surgical experiment, rats were given morphine (2 mg/Kg) for pain relief after anesthesia. The other end of a single-cavity perfusion tube was attached to a continuous-perfusion pump and was orally put in the oesophagus, fixed 2–3 cm above the oesophagus and stomach junction. Subsequently, for 50 minutes, 10 mL/h of 0.1 mol/L hydrochloric acid (KDX007; Shanghai Kehua Bio-Engineering Co., Shanghai, China) was dropped. Finally, in the SJHG group, at week 3, a gastric gavage was performed with SJHG granular solvent (4 g/kg, the human-equivalent dose) instead of normal saline, while the rest of the process was the same as that in the NERD group. During the experiment, the rats' water intake, hair, and emotional condition were all monitored. Finally, the rats were slaughtered, and substantial pieces of their brains, oesophagus mucosa, and spinal cord were removed for further research.

### 2.3. Transmission Electron Microscopic Observation

Tissue blocks of ≤1 mm3 diameter were immediately cut from the rats' spinal cord and oesophagus after they had been slaughtered by a sharp blade within 1-3 minutes. These blocks were further transferred to an Eppendorf tube containing freshly prepared TEM fixative (G1102, Servicebio, Wuhan, China) for further fixation at 4°C for preservation and transportation before being placed in an ice bath for preservation and transportation. Post-fixation, the tissues were maintained away from light in PB with 0.1 M concentration (pH 7.4) containing 1% OsO_4_ at room temperature for 2 hours. The tissue samples were then rinsed thrice with PB after OsO_4_ removal for 15 minutes each time.

Using acetone as an intermediate solvent, the dehydration of fixed tissue samples was performed in an ethanol series before being embedded in EMBed 812 resin (90529-77-4; SPI). Furthermore, these resin blocks were cut to a thickness of 60–80 nm using an ultra-microtome (UC7; Leica, Wetzlar, Germany). Afterwards, ultra-pure water was used to rinse thrice with 2% uranium acetate saturated alcohol solution and 2.6% of lead citrate to avoid light and CO_2_ staining for 8 minutes. The cuprum grids were initially dried through filter paper and then placed on the grids board to dry overnight. The dried grids were further visualized through a transmission electron microscope and obtained results were saved in image format.

### 2.4. Immunohistochemical Analysis

Additionally, for histochemistry analysis, 4 m slices of the paraffin tissue block were cut. The c-fos (cat. #11069.1 : 500; Servicebio) antibody drips were prepared in a specific proportion with phosphate-buffered saline on the blocks and incubated overnight at 4°C. The tissue was coated with a secondary antibody that was horseradish peroxidase- (HRP-) labeled (HRP-labeled goat anti-rabbit, cat. #G23303.1 : 200; Servicebio). An automated image analysis system (Servicebio, Wuhan, China) was used to read the tissue measurement area. This system divided the positive grade as 0, 1, 2, and 3 points for without staining, weak positive light yellow, medium positive tan, and strong positive tan, respectively. On the immunohistochemistry slices, these images were obtained employing a tissue slice digital scanner.

### 2.5. TMT Proteomics

Before being placed into a 5 mL centrifuge tube, the tissue sample was pulverized into cell powder using liquid nitrogen. The cell powder was then sonicated thrice on ice with a four volume of lysis buffer (8 M urea, 1% protease inhibitor cocktail) using a high-intensity ultrasonic processor (Scientz, Ningbo, China). The remaining debris was removed by centrifugation at 12,000 g for 10 minutes at 4°C. Finally, the supernatant was collected, and the protein content was measured using a bicinchoninic acid kit, as directed by the manufacturer.

The protein solution was reduced with 5 mM dithiothreitol for 30 min at 56°C whereas was alkylated with 11 mM iodoacetamide for 15 min at room temperature in darkness for digestion. After that, the protein sample was diluted by adding 100 mM TEAB to a urea concentration of <2 M. Finally, trypsin was added at 1 : 50 and a 1 : 100 trypsin-to-protein mass ratio for the overnight and 4 h digestion, respectively. The peptides were then desalted using a C18 SPE column.

The tryptic peptides were first dissolved in 0.5 M of TEAB before being used. After each peptide channel had been tagged with its appropriate TMT reagent (Thermo Fisher Scientific), it was incubated for 2 h at room temperature. For determining the labeling efficiency, five mL of each sample were desalted, pooled, and evaluated via mass spectrometry (MS). Following the evaluation of labeling efficiency, samples were quenched with a 5% hydroxylamine solution. Subsequently, the pooled samples were desalted and dried through Strata X C18 SPE column (Phenomenex, Torrance, CA, USA) and vacuum centrifugation.

The peptides were separated on a 300 Extend C18 column (5 m grain size, 4.6 mm inner diameter, 250 mm length; Agilent Technologies, Santa Clara, CA, USA) using high-pH reversed-phase high-performance LC. The setting for the procedure was set at 9 pH, 8%–32% acetonitrile as the peptide gradient. The 60 components were separated in 1 h, and the peptide was then consolidated into nine components and freeze-dried in a vacuum for future procedures.

The peptides were separated using the EASY-NLC 1200 ultra–high–performance LC system (Thermo Fisher Scientific) after being dissolved by mobile phase A (aqueous solution 2% acetonitrile and containing 0.1% formic acid). The mobile phase was prepared in an aqueous solution having 90% acetonitrile and 0.1% formic acid. The procedure for establishing a liquid-phase gradient was as 7%–22%; 22%–32%; 32%–80%, and 80% B from 0 to 40, 40 to 53 min, 53 to 57 min, 57 to 60 min, respectively. The flow rate remained constant at 500 nL/min. The peptides were separated using an ultra-high-performance liquid-phase system before being fed into an NSI ion source and analyzed with the Q-EXactive HF-X mass spectrometer (Thermo Fisher Scientific). The ion source voltage was set to 2.1 kV, and the peptide parent ions and secondary fragments were identified and analyzed using the high-resolution Orbitrap system. The first- and second-level MS scanning ranges were set as 350–1600 m/z, and 100 m/z, with a scanning resolution of 120,000 and 30,000, respectively. Following the completion of the first level of scanning, the parent ions of the top 20 peptide segments in terms of signal strength were selected to enter the high-energy collision dissociation (HCD) collision cell in sequence. During the data-collection mode, they were splintered using 28% of the fragmentation energy. Similarly, the MS analysis at the second level was carried out in this sequence. To reduce the number of times that parent ions were repeatedly scanned, the automatic gain control was set to 1E5, the signal threshold was set to 8.3E4 ions/s, the maximum injection length was set to 60 ms, and the dynamic exclusion period of the MS/MS scan was set to 30 seconds.

The MaxQuant search engine (version 1.6.15.0) was used to carry out the processing of the MS/MS data that was produced. These are the settings for the retrieval parameters: the database that was utilized was Rattus norvegicus 10116 PR 20210721.fasta (29934 items), and the reverse database was included so that the false-positive rate that is produced by random matching may be determined. A common contamination database has been introduced to the database to reduce the impact of contaminated proteins on the identification findings of the proteins under investigation. Trypsin/P was chosen as a cleavage enzyme because it allows for up to two missed cleavages to occur. Mass tolerance for precursor ions was set at 20 ppm in the first search and 5 ppm in the main search, while mass tolerance for fragment ions was set at 0.02 Da. The bacterial carbamidomethylation of Cys was characterized as a fixed change, whilst the acetylation of the protein's N-terminal and the oxidation of Met were, respectively, regarded as changeable alterations. The percentage of cases involving false positives has been brought down to 1%.

### 2.6. Bioinformatics Analysis

Moreover, the UniProt-GOA database (http://www.ebi.ac.uk/GOA/) was accessed to retrieve the Gene Ontology (GO) annotation proteome. The IDs were transferred to detected proteins via UniProt identifiers and further mapped to GO identifiers based on the protein identifier. All protein GO functions were annotated using InterProScan for those proteins that failed to be annotated through the UniProt-GOA database. Furthermore, GO annotation for proteins was characterized based on their molecular function, biological process, and cellular component. Additionally, the clustering functional characterization of homologous proteins was performed. The COG (cluster of orthologous groups) refers to the protein lineal homologs in COG/clusters of orthologous groups for eukaryotic complete genomes (KOG) function. COG is a database maintained by the NCBI and classified into two categories: prokaryotes (COG database) and eukaryotes (KOG database). Database evaluation and analysis were used to compare and analyze DEPs for COG/KOG functional classification. It was discovered that proteins in eukaryotic tissue cells may attach to certain types of membranes, which allowed to map them to specific parts of the cell. Therefore, the WolF Psort program was used to annotate the proteins' subcellular locations in the cytoplasm, Golgi apparatus, nuclear matrix, extracellular region, endoplasmic reticulum, ribosome, and vacuole, mitochondria, nucleus, peroxisome, and cytoskeleton.

A protein domain is a segment of a protein with a conserved sequence that can operate independently in most cases. It is made up of 25–500 amino acids and is the structural component of molecular function. These regions are small in size, have a stable structure, and can be folded into functioning structures independently. A domain may be found in numerous proteins, and a domain can be found in multiple proteins. Protein-domain annotation was done for identified proteins in the project data using the Pfam database and the PfamScan program. Protein pathways were annotated using the Kyoto Encyclopedia of Genes and Genomes (KEGG) database. The KAAS server of KEGG was employed to annotate proteins whereas the KEGG mapper was accessed to map the annotation result onto the KEGG pathway database. The bubble plot revealed a considerable enrichment of these annotated DEPs.

At least one ≥1 functional classification substantially enriched in the proteome was filtered out (*P* < 0.05) using GO functional classification information and *P*-value enrichment of the related proteome. The chosen *P*-value data matrix was first changed using the −log10 logarithm transformation, and further categorization of different functions was performed through Z transformation. Finally, for unilateral clustering analysis, the hierarchical clustering approach was applied. Additionally, the association among clusters was highlighted as a heat map generated through a heatmap.2 function from the R package. The horizontal heat map depicts the results of various groups' enrichment tests, while the vertical heat map depicts the description of differentially expressed enrichment-related functions. The degree of enrichment is shown by the DEPs in distinct categories and the accompanying color blocks of functional descriptions such as red and blue color indicate the high and low levels of enrichment.

PPIs were found by searching all DEP sequences or accessions against the STRING (version 11.5) database. Only interactions between proteins in the search data set were used to exclude external candidates. We used STRING's “confidence score” metric to find all interactions with a “high confidence” value of ≥0.7. Subsequently, the R tool networkD3 was used to display the STRING PPI network.

### 2.7. Statistical Analysis

The processing and analysis of obtained data were carried out using SPSS 17 (IBM Corporation, Armonk, NY, USA). It was determined to express the measurement data in terms of the mean ± standard error of the mean values. To compare the features of the samples between the two groups, Student's *t*-test was utilized. *P* < 0.05 was considered a statistically significant cutoff.

### 2.8. Verification by Western Blot Analysis

An assay buffer (G2002; Servicebio) was used to extract protein from the Cingulate Gyrus and Spinal Dorsal Horn nerve tissue, and the bicinchoninic acid protein assay (G2026; Servicebio) was used to measure the concentration of proteins. To separate the same number of proteins and transfer them to a polyvinylidene difluoride membrane, we used an SDS-PAGE gel (S8010-500g; Solarbio) electrophoresis. This membrane was incubated overnight with the corresponding primary antibody (anti-kininogen 1 [Kng1]: cat.#DF6544, 1:1000 from Affinity Biosciences, Cincinnati, OH, USA; anti–junctional adhesion molecule A [JAM-A]: cat#DF63731:1000 from Affinity Biosciences; and anti-*β*-actin cat.#GB15001, 1:2000 at 4°C from Servicebio), further incubated with HRP-conjugated secondary antibody (cat.#GB25301,1:5000; Servicebio). After chemiluminescence treatment, Photoshop (Adobe, San Jose, CA, USA) and Alpha (AlphaEase FC, version 6.0.0) software processing were used to analyze the optical density of the film.

## 3. Results

### 3.1. Rats' General Health State

There were no fatalities in the control group throughout the trial; however, two rats died in the model group and three rats died in the SHJG group. Each group of rats had a healthy mental condition, lustrous hair, and typical drinking behavior prior to modeling. Rats in groups other than the normal group exhibited a weaker mental state, lower feeding and drinking habits, and yellow and withered hair, and were more irritable when the stressor was administered. At the end of the 28th day, the weights of rats in the normal and model groups were statistically substantially different, with the normal group being heavier (*P* < 0.05, see Table 2).

Note: ∗*P* < 0.05; ^#^*P* > 0.05, compared to the normal group.

### 3.2. VH and NERD Signs

Changes in esophageal epithelial cells and the synaptic cleft of the spinal cord dorsal horn were observed by TEM. Under 2.5-K electron microscopy, the NERD group's epithelia had much wider intercellular gaps than those in the control group (see Figure 1(a)). Synaptic vesicles in the spinal dorsal horn of rats in the NERD group increased under the 15-K electron microscope compared to those in the NC and SJHG groups (see Figure 1(b)).  Figure 1(c) shows the immunohistochemical outcomes. The content of c-fos in the spinal cords of rats in the NERD group was higher (*P* < 0.0001) than in the NC group, according to the integrated optical density. Meanwhile, the SJHG group's c-fos content was substantially reduced (*P* < 0.0001) as compared to the NERD group. The NERD with VH model caused by stress was also validated by these data.

### 3.3. Sample Quality Control

SDS-PAGE electrophoresis was performed to evaluate the protein's quality control.  Figure 2(a) shows that the protein bands were clean, homogeneous, and free of degradation, indicating that they would be suitable for use in the experiment. The reproducibility of protein quantification was evaluated using the RSD technique. Smaller RSD values indicate better quantitative repeatability. The RSD was found to be <10%, showing that the quantitative technique was accurate and consistent (see Figure 2(b)).

### 3.4. LC-MS/MS Analysis

MS was used to produce 302,667 secondary spectrograms for the current study. After examining the protein theory database, 92,229 valid mass spectrograms were discovered, with a 30.47% usage rate. A total of 52,851 peptides were found using spectrographic analysis, with 47,528 of them being specific. A total of 6,982 proteins were discovered, with 6,003 of these being measurable (see Figure 3(a)). Consequently, only 64 differentially expressed proteins were predicted with the cutoff criterion set as fold change = 1.2 and *P* < 0.05, including 38 upregulated proteins and 26 downregulated proteins (see Figures 3(b) and 3(c)).

### 3.5. Functional Classification of DEPs

GO functional categorization revealed that the differential molecules were mostly involved in cellular activities, biological control, metabolic processes, reaction to stimuli, immune system processes, and biological adhesion (see Figure 4(a)). Secondary metabolite production, transport and catabolism, chromatin structure and dynamics, transcription, and signal transduction pathways were all implicated in these differentially expressed molecules according to the COG/KOG categorization system (see Figure 4(b)). DEPs were found in the nucleus in 35.94% (*n* = 23) of the samples, in the cytoplasm in 20.31% (*n* = 13), and in the extracellular space in 18.75% (*n* = 12) of the samples. In addition to mitochondria and plasma membranes, there were others (see Figure 4(c)).

### 3.6. DEPs Protein Domains and Pathway Enrichment Analysis

Bubble plots were used to show protein domains and KEGG pathway enrichment. DEP enrichment was shown in the image by the circles. DEP enrichment is very significant (*P* < 0.01) in red, significant (*P* > 0.05) in yellow, and nonsignificant (*P* < 0.05) in blue. The fold enrichment is represented by the size of the circle. The components of DEPs centered on the complement Clr-like EGF-like, cystatin domain, core histone H2A/H2B/H3/H4, and calcium-binding EGF domain, according to protein-domain enrichment analysis. Systemic lupus erythematosus, neutrophil extracellular trap formation, complement and coagulation cascades, African trypanosomiasis, necroptosis, alcoholism, Chagas disease, inflammatory mediator–regulation of TRP channels, neuroactive ligand-receptor interaction, and sphingolipid signaling pathway were identified as significant enrichment signal pathways of DEPs by KEGG analysis (see Figure 5).

### 3.7. DEPs Cluster Analysis

DEPs were classified into four categories based on the AF/SR ratio (Q1, 0.769, Q2, 0.769–0.833, Q3, 1.2–1.3, and Q4, > 1.3). (see Figure 6). Q3 and Q4 constitute the majority of upregulated proteins, and these proteins were localized in the nucleus and organelle lumens of the cell (see Figure 6(c)) and primarily various epigenetic regulatory molecules (e.g., histone H2A, histone H2B, ribonucleoprotein complex, nuclear factor 1) (see Figure 6(d)). The proteins that were downregulated (Q1) were mostly localized in the extracellular compartment involved in the negative control of biological immune responses and the activation of associated proteins. The molecular function of downregulated proteins is mainly to bind with a variety of metal ions and regulate the activity of peptidase inhibitors and endopeptidase inhibitors (see Figures 6(b)–6(d)).

### 3.8. PPI Network Analysis of DEPs

We generated a PPI network of the differential proteins to better illustrate the interrelationships between them. Circles with green DEPs and red DEPs indicate DEPs, which are the proteins that have been downregulated. The results showed that there were six important node proteins, as follows: kininogen-1 (Kng1, F7EUK4), four nodes; T-Kng1 (Map1, P01048), four nodes; histone H2B (Hist3h2bb, M0RBQ5), four nodes; proenkephalin-A (Penk, P04094), four nodes; pro-MCH (Pmch, G3V6L0, CPB1), three nodes; and fibrillin 1 (Fbn1, G3V9M6, TTR), three nodes (see Figure 7).

### 3.9. Validation of the Differently Expressed Proteins by Western Blotting

Figure 8 shows that compared to the NC group, the Kng1 protein level in the cingulate gyrus increased in the NERD group, while the JAM-A protein level did not change significantly. Moreover, the SHJG group's JAM-A protein level increased significantly in comparison to the NERD group, while the Kng1 protein level decreased.

## 4. Discussion

There is mounting evidence to support the idea that VH plays a significant part in the etiology of NERD; nevertheless, the research that has been conducted so far on VH has not been sufficient, such as by providing an explanation for why VH causes mental abnormalities. We found that the proteomics of brain tissue in NERD has not been studied yet, which is crucial for understanding the pathogenesis of NERD. However, the effects of NERD on brain tissue may be multifaceted and complex, which may lead to a significant decrease in the accuracy of prediction. According to TCM, NERD is mainly caused by “ liver qi stagnation, stomach discomfort, and adverse rising of the stomach qi” [20]. At the same time, TCM believes that VH and function of “liver” are closely related [21]. Therefore, we choose to treat liver depression, qi stagnation of traditional Chinese medicine formula for research.

We confirmed whether the disease model was successfully established by TEM and IHC analysis. After induction of emotional stress, the c-fos protein level and synaptic vesicle release increased in the dorsal horn of the spinal cords of rats but decreased after treatment with SHJG. This indicated that splanchnic hypersensitivity was observed in NERD model rats and that this central nervous sensitivity could be improved by SHJG. In addition, the esophageal mucosa of rats was observed by TEM, and the DIS in the esophageal submucosa was confirmed in NERD model rats. SJHG's validity was proven by the aforementioned findings, which showed that the NERD model had been effectively created.

To further understand the mechanism by which SJHG improves VH in brain tissue, we analyzed the molecular profile of rat cingulate gyrus tissue using a TMT proteomics system and found 64 proteins with distinct expression differences. We discovered that these differentially expressed molecules in the nucleus, extracellular area, and cytoplasm were linked to biological regulation, cellular processes, metabolic processes, stimulus response, immune system processes, and biological adhesion through classification and functional enrichment analysis. In addition, four of the ten significant signaling pathways, including systemic lupus erythematosus, neutrophil extracellular trap formation, inflammatory mediator–regulation of TRP channels, and complement and coagulation cascades, were associated with the immune system. The transmission of brain signals is mediated by three pathways: inflammatory mediator–TRP channel regulation, neuroactive ligand-receptor interaction, and the sphingolipid signaling route. Other signal pathways include necroptosis, alcoholism, Chagas disease, and African trypanosomiasis. The differential molecules involved include Kng1, JAM-A, phosphatidylinositol 3-kinase regulatory subunit beta (Pik3r2), complement component C9, Map1, Penk, and histone H2A. These results suggest that SJHG may improve VH by regulating the inflammatory response of brain tissue or by inhibiting the abnormal activation of various nerve cells. We discovered six critical hub proteins, each with ≥3 nodes, using PPI network analysis. By analyzing the differential proteins in the network, we found that five differentially expressed histones in the network were involved in DNA modification, affecting epigenetic inheritance. In addition, we found interactions between some immune-associated molecules and molecules related to neuroactive ligand–receptor interaction, such as Kng1, Pmch, Hrg, Map1, and Penk. These results suggest that SJHG treatment of VH may be accomplished by influencing the interaction between the immune and nervous systems. At the same time, these regulatory effects may be accomplished through histone modifications.

Through a bioinformatics analysis and literature review, we found that Kng1 and JAM-A proteins might be related to the mechanism of VH, so we verified the proteomics results by WB and confirmed that Kng1 and JAM-A protein levels had significant changes. Kng1 was significantly upregulated in the NERD group, while SJHG could restore Kng1 protein expression to normal levels. Meanwhile, JAM-A protein levels were upregulated in the NERD group and SJHG group.

High- and low-molecular-weight Kng (HMWK and LMWK) are two proteins with distinct structures that may be produced by varied shearing in the presence of a Kng1 protein [22]. HMWK, as a precursor protein of the kallikrein–kinin system (KKS), is essential for the maintenance of the functional stability of the KKS [23, 24]. Composed of proteolytic enzymes and biogenic peptide cascades, KKS is widely distributed throughout the brain and is involved in the progression of various neurological diseases [24]. On the other hand, HMWK can release bradykinin after enzymatic catalysis to reduce the hypersensitivity of pain in nerve pain model rats [25]. These consequences propose that the abnormal expression of Kng1 may be a cause of VH in rats with NERD disease, and SJHG may treat NERD by reducing Kng1 [26]. JAM-A is a kind of adhesion protein containing a PDZ domain on its cell membrane. Currently, JAM-A is found in the nerve, epithelium, endothelium, and blood cells. It crosses the cell membrane and is divided into two parts: extramembrane and intramembrane. The extramembrane portion of JAM-A acts as a “fence” that regulates cell adhesion and migration [27, 28]. JAM-A is an important protein that constitutes the tight junction between cells, which maintains the integrity of the blood–brain barrier and prevents inflammatory factors from entering the brain through this barrier [28, 29]. Moreover, adhesion receptors on adjacent cells can adapt to changes in the microenvironment because of the information conveyed by adhesion receptors on their cells. Adhesion receptors use their cytoplasmic domains (including FERM, proline-rich motifs, PDZ domains, and phosphorylation sites) to bind to appropriate specific interaction motifs in cytoplasmic proteins and transmit intercellular signals [30–32]. SJHG's therapy of VH may be based on the hypothesis that JAM-A expression is being increased.

Finally, in this study, SJHG reduced the expression level of Pik3r2, which was of interest to us. Pik3r2 is a protein that is involved in the PI3K/Akt signaling pathway, which is a signaling pathway that has been implicated in the proliferation and survival of neurons in the central nervous system [33, 34]. Indirectly, the PI3K/Akt signaling system regulates autophagy, resulting in the PI3K/Akt signaling pathway associated with neuronal survival [35]. This route is used by a variety of neuroendocrine substances to exhibit neuroprotective effects, such as brain-derived neurotrophic factor (BDNF). The PI3K/Akt signaling pathway is important in the development of cognitive capacities as well as the maintenance of synaptic plasticity in studies [36–38]. SJHG therapy for VH seems to be associated with alterations in the PI3K/Akt signaling pathway in the rat's cingulate gyrus, according to the findings of this study.

## 5. Conclusions

In the cingulate gyrus of NERD rats, SJHG treatment altered the expression levels of several proteins. The differential molecules involved include Kng1, JAM-A, Pik3r2, complement component C9, Map1, Penk, and histone H2A. And these molecules were significantly enriched in immune response and the transmission of neural signals. These results suggest that SJHG may improve VH by regulating the inflammatory response of brain tissue or by inhibiting the abnormal activation of various nerve cells. These results provide new evidence of SJHG treatment of NERD by ameliorating VH. In addition, we found two therapeutic targets of SJHG—namely, Kng1 and JAM-A. And SJHG may influence autophagy through the PI3K/Akt signaling pathway. However, there are some shortcomings of this study. SJHG is a compound preparation. Although possible targets of action were found, it cannot explain what specific components play a role and cannot clarify the specific mechanism of action. Relevant experiments were not performed to verify that SJHG affects the PI3K/Akt signaling pathway. There may be discoveries in NERD diagnosis and treatment utilizing vast numbers of samples and in-depth mechanism studies of the molecules uncovered by this work, even if they are not yet understood how well these differential molecules are involved in the pathogenic processes of VH.

## Figures and Tables

**Figure 1:** Electron microscopy and immunohistochemical results. (a) Intercellular spaces of epithelia of the esophageal mucosa as observed by TEM (×2.5 K). (a. NC group, b. NERD group; black arrows indicate the interstitial space). (b) Synaptic vesicles as observed by TEM (×15 K). (c. NC group, d. NERD group, e. SJHG group; black arrows indicate synaptic vesicles). (c) Expression of c-fos protein in the spinal cords of rats (immunohistochemical staining, ×200) (f. group, g. NERD group, h. SJHG group). (d) IOD values of c-fos protein in the spinal cord of rats in the 3 groups. ∗∗∗∗*P* < 0.0001, compared with the NERD group.

**Figure 2:** Quality control of the samples. (a) SDA-PAGE diagram. (b) Protein RSD distribution between repeated samples. Note: N means model group, T means SJHG group.

**Figure 3:** Results of the LC-MS/MS study. (a) MS data fundamental statistics. (b) DEP quantity dispersion. (c) DEPs volcano diagram.

**Figure 4:** Functional annotation of DEPs. (a) GO term's function annotations. (b) COG/KOG function. (c) DEPs localization in subcellular compartments.

**Figure 5:** (a) KEGG pathways of DEPs. (b) Protein domains of DEPs.

**Figure 6:** Cluster analysis of GO functional enrichment of DEPs. (a) The distribution of DEPs in Q1–Q4. (b) Biological processes. (c) Cell composition. (d) Molecule function.

**Figure 7:** The network of protein-protein interactions that occur between the different proteins.

**Figure 8:** Protein expressions of JAM-A and Kng1 among the groups. The expression level of JAM-A and Kng1 were analyzed through western blot analysis. ∗∗∗*P* < 0.001, ∗∗*P* < 0.01, ∗*P* < 0.05.

**Table 1:** Components of SJHG.

Latin name	Chinese name	Amount used
Radix Bupleuri	Chaihu	9 g
Cyperi Rhizoma	XiangFu	9 g
Arum Ternatum Thunb	BanXia	12 g
Citrus Reticulata	ChenPi	12 g
licorice	GanCao	9 g
Inulae Flos	XuanFuHua	9 g
Aurantii Fructus	ZhiQiao	12 g
Reddle	DaiZheShi	30 g
Scutellariae Radix	HuangQin	10 g
Chuanxiong Rhizoma	ChuanXiong	9 g

**Table 2:** The average weight (g) of rats belonged to the normal group and the model group ($\bar{x}\pm s$).

Group	Baseline	14th day	28th day
Normal	270.33 ± 13.05	325.67 ± 12.00	365.25 ± 16.98
Model	275.00 ± 9.682^#^	327.09 ± 10.45#	333.8 ± 16.61∗

## Data Availability

The labeled dataset used to support the findings of this study is available from the corresponding author upon request.
